# Bitterness intensity prediction of berberine hydrochloride using an electronic tongue and a GA-BP neural network

**DOI:** 10.3892/etm.2014.1614

**Published:** 2014-03-11

**Authors:** RUIXIN LIU, XIAODONG ZHANG, LU ZHANG, XIAOJIE GAO, HUILING LI, JUNHAN SHI, XUELIN LI

**Affiliations:** 1 Department of Pharmacy, The First Affiliated Hospital of Henan University of Traditional Chinese Medicine, Zhengzhou, Henan 450000, P.R. China; 2 College of Pharmacy, Henan University of Traditional Chinese Medicine, Zhengzhou, Henan 450008, P.R. China

**Keywords:** electronic tongue, genetic algorithm-back-propagation neural network, bitterness intensity, bitterness prediction model, berberine hydrochloride

## Abstract

The aim of this study was to predict the bitterness intensity of a drug using an electronic tongue (e-tongue). The model drug of berberine hydrochloride was used to establish a bitterness prediction model (BPM), based on the taste evaluation of bitterness intensity by a taste panel, the data provided by the e-tongue and a genetic algorithm-back-propagation neural network (GA-BP) modeling method. The modeling characteristics of the GA-BP were compared with those of multiple linear regression, partial least square regression and BP methods. The determination coefficient of the BPM was 0.99965±0.00004, the root mean square error of cross-validation was 0.1398±0.0488 and the correlation coefficient of the cross-validation between the true and predicted values was 0.9959±0.0027. The model is superior to the other three models based on these indicators. In conclusion, the model established in this study has a high fitting degree and may be used for the bitterness prediction modeling of berberine hydrochloride of different concentrations. The model also provides a reference for the generation of BPMs of other drugs. Additionally, the algorithm of the study is able to conduct a rapid and accurate quantitative analysis of the data provided by the e-tongue.

## Introduction

Taste-masking, particularly bitterness taste-masking, is an important issue that pharmaceutical scientists encounter. Studies on methods of quantifying bitterness intensity and the factors contributing to bitterness generation are likely to aid pharmaceutical workers conducting taste-masking research.

The fundamental quantitative method for determining bitterness intensity is the traditional human taste panel method (THTPM) (1). In the present study, the bitterness intensity obtained by the THTPM is designated the human taste bitterness intensity (I*_h_*). According to the different determination approach, I*_h_* is divisible into rank bitterness intensity (I*_0_*) and relative bitterness intensity (I*_1_*). The THTPM is widely used in the fields of food (2), functional food (3) and drugs (4,5). However, the subjectivity of the THTPM is marked and its operation is complicated. It is possible to collect various types of chemical information about drug solutions through sensors using an electronic tongue analyzer (e-tongue) (6,7), and then based on known information, such as the taste information provided by the THTPM, the bitterness intensity, sweetness-sugariness intensity and other taste information may be identified through certain mathematical methods. The bitterness intensity obtained by this method is known as the e-tongue bitterness intensity (I*_e_*) in the present study. This method has numerous advantages, including quantified data, stable output and no potential safety risk, which compensates for the deficiency of the THTPM (8). The e-tongue system has been developed for the taste measurement of bitter drug substances in accurate taste comparisons for the development of palatable oral formulations (9). The e-tongue is a useful tool in pharmaceutical development for the qualitative and quantitative evaluation of drug substance taste, as well as bitterness masking efficiency, without performing laborious gustatory sensation tests in humans (10).

In order to analyze the e-tongue data and predict the gustatory sensation of a sample accurately and reliably, the analysis should be based on instructional learning methods such as partial least squares (PLSs) and support vector machines. In addition, an accurate and reliable bitterness prediction model (BPM) (10–12) should be set up between e-tongue sensing information and I*_h_*, to incorporate the results of the THTPM. Only in this way is it possible to achieve the precise prediction of the bitterness intensity of a drug. Different machine learning methods have different characteristics. For example, PLS is a linear method, although it has its advantages (simple, accurate and stable), while back-propagation neural networks (BPNNs) have fine non-linear mapping ability, but their algorithms easily fall into the local extreme point (12). Genetic algorithms (GAs), which imitate the inheritance and evolution of creatures in the physical environment, are grading-up probabilistic searching algorithms that adapt to the overall situation and overcome the disadvantages of BPNNs. There are a variety of ways to combine a GA and a BPNN (GA-BP), including the application of the GA to increase the optimization of the initial weight and offset of the BP network (13–15). To the best of our knowledge, studies of a BPM built using this method have never been reported.

Berberine hydrochloride is the essential component of the traditional Chinese medicine Rhizoma Coptidis, and it is also a popular antibacterial agent (16). Due to its high bitterness intensity, it is usually used as a reference material in studies concerning the taste-masking of bitter drugs. The present study demonstrates a method of using various concentrations of berberine hydrochloride solution as the investigative support in the analysis of the results of an e-tongue and the THTPM. In addition, the prediction of the I*_0_* of berberine hydrochloride was achieved using the GA-BP to establish its BPM.

## Materials and methods

### Volunteer screening

Strict screening including bitter taste sensitivity was conducted to recruit volunteers and 20 healthy volunteers were selected as the subjects (nine male and 11 female). This study was conducted in accordance with the Declaration of Helsinki and with approval from the Ethics Committee of the First Affiliated Hospital of Henan University of Traditional Chinese Medicine (Zhengzhou, China). Written informed consent was obtained from all participants.

### Concentration selection of the reference samples and sample preparation

According to literature methods (1,17,18), a scale of 1–5 was used to determine the bitterness intensity, and each score on the scale was assigned a certain bitterness distance which corresponded with a certain concentration. The concentration was obtained by pre-testing of the berberine hydrochloride reference solution (lot number, 101002; Sichuan Province Yuxin Pharmaceutical Co., Ltd., Chengdu, China) with different concentrations by the subjects (Table I).

### Preparation of the test samples

The berberine hydrochloride was formulated to various concentrations (0.001, 0.0025, 0.01, 0.025, 0.1, 0.25, 0.5, 1 and 2.5 mM) which were referred to as S1–S9, respectively.

### Standardization between the taste evaluation of the subjects and the bitterness values of the reference sample groups

According to the method of Kawano *et al* (18), the subjects took 20 ml reference solution at various concentrations in a tasting cup, held the aforementioned reference solutions in their mouth for 15 sec and were informed of the bitterness scale and bitterness intensity. Following tasting of the sample, the subjects gargled well and waited for at least 15 min prior to tasting the subsequent sample.

### Gustatory sensation evaluation of test samples

Following the previously described procedure, the subjects evaluated and provided a numerical value for test samples according to their taste sensation and the bitterness scale of the reference solutions. The results were assigned on designed evaluation forms. Subsequently the subjects gargled well and waited for at least 15 min prior to tasting the subsequent sample.

### Outlier handling

In this study, the subjects may have individual differences and several outliers emerged among the experimental data. The outliers were tested and removed using the Grubbs’ testing method. Only one outlier was removed in each cycle. Oversized and undersized outliers may exist in taste experiments, so the statistical tests used in this study were two-sided. The significance and rejection levels were set as 0.1 and 0.05, respectively.

### Determination of e-tongue data

E-tongue and data acquisition experiments were performed using an Astree II electronic tongue (Alpha M.O.S, Toulouse, France). The e-Tongue was capable of discriminating between substances with different tastes, and the sensors appeared to be cross-selective for five basic tastes: Sourness, sweetness, bitterness, saltiness and umami. A strong linear correlation between berberine hydrochloride bitter and concentration has been observed in the concentration range 0.93 18.63 mg/l. (19).

With regard to the nine concentrations of berberine hydrochloride solution, the sensors were rinsed with deionized water in six beakers of water for 10 sec following each pre-test. The sensors were rinsed well prior to analyzing the samples. The sample (80 ml) with each concentration was placed into a 120-ml beaker used specifically for the e-tongue and the beaker was placed on an automatic sampling plate. All samples were analyzed seven times and each analysis cycle lasted 120 sec. For these experiments, the samples were analyzed at room temperature, and only the last 120 sec of data were used in the analysis. Samples were replicated seven times, with only the last four replications used in mathematical processing and analysis.

### Processing of the GA-BP

This study utilized the application of a GA to optimize the initial weight and offset of the BPNN. The main process of the algorithm was divided into two stages: i) On the basis of the initialization model, the connection value was encoded and the BPNN offset to compose the chromosomes of the GA, the chromosomes were optimized by the GA and the decoded chromosomes were assigned to a neural network; and ii) the network weight was further optimized and was offset by the local optimization ability of the training function of the BP. The flowchart is shown in Fig. 1 and the functions in the dotted box constitute the first stage.

### Model initialization and parameter selection

The vectors of the BPNN, which used A, B, Z_1_ and Z_2_ as input vectors and Y as the output vector, were normalized in the range [−1,1] to eliminate the effects of dimension. Three-layer structures which included a hidden layer were selected through pre-testing and intra-checking. The node point of the hidden structure was five; the transfer functions were tansig and purelin; the training function was traingd; the learning rate was 0.05; the target error was 10^−4^; and the maximum number of training cycles was 18,000.

The GA adopted a real coding pattern to arrange the 46 parameters of the BP network, the connection values of which were included with definite order. The aim was to compose the chromosomes of the GA. The population was 50 and the genetic algebra was 500. The difference between the original output vector normalization and the non-normalized prediction output vector was defined as the residual; therefore, the fitness function was the reciprocal of the sum of squared residuals. According to the ranking selection method of normal geometric distribution, q was 0.08, which determined the probability selection table. Taking arithmetic crossover, the frequency of evolutionary crossover in every generation was two. Namely, crossover operation of individual accounts for the largest proportion of population (50) 4%. By adopting the non-uniform mutation operator, the shape parameter b was calculated to be 3. The frequency of mutation operation with each individual mutation probability being 0.053 was four times in each generation of evolution.

### Training and establishment of the model

Certain GAs after 500 generations of evolution did not meet the GA target precision of 10^−3^, and the best individual was assigned to the BP network.

### Optimization and evaluation of the model

The jackknifing cross-validation method was used for the optimization and evaluation of the model. In order to avoid the result information of the parallel determination distributing in the training set and validation set at the same time, thus causing high fitting of the error model, each reserved verification set was unified into four-fold parallel test results of each sample in the design process.

The root mean square error of cross-validation (RMSECV) and the correlation coefficient (R) between the true and predicted values in cross-validation are regarded as the evaluation indices. The formula for calculating R omitted slightly. The formula for calculating RMSECV was as follows: RMSECV = √[∑(*I_0i_* *- Î_0i_* *)^2^/n]*, where *n* is the total number of observations; *I_0i_* is the corresponding I*_0_* of the *ith* observation; and *Î_0i_* is the prediction value of I*_0i_* obtained from the model which was established using the rest of the n-4 observations by removing the *ith* observation.

When conducting the cross-validation, owing to the algorithm including standardization and reverse standardization processing steps, the two ends of the data (eight groups of data with the maximum and minimum bitterness) were in processing beyond the scope of normal values, causing greater errors; and model prediction was not sharply extended to the two ends when forecasting the model. Therefore, the following data are the results that were obtained following the removal of the data from the two sides of the forecasting results. In addition, on account of the randomness of the initial value, six groups of cross-validation results were calculated. Modeling was carried out with all the data as a training set.

### Comparison with other modeling methods

The same e-tongue data may be modeled using multiple linear regression (MLR), PLS regression and artificial neural networks for comparison with the results generated by the GA-BP model. Processing of the data was conducted with cross-validation and modeling with the GA-BP method. In PLS regression, the RMSECV and R of cross-validation between the true and predicted values for an index are utilized to optimize the number of latent variables. The artificial neural network opted for the same parameters as the GA-BP.

## Results

### Bitterness intensity order of the I_0_ taste results

Following processing of the experimental data, the results showed that 1.2 in data group 1 and 2.6 in data group 3 were deviation value, scilicet it reached the detectable level (α=0.05), but not to the eliminate level (α=0.01), so were retained. No data were eliminated in this experiment. Samples of nine concentrations and their corresponding bitterness intensity order are shown in Fig. 2. There are 36 groups of data for the BPM in total, and each group contains seven root sensor responding values, so this model has a total of 36 × 7 (252) data.

### Training and establishment of the model

Fig. 3 shows the maximum fitness and the change of the average fitness of the groups in the evolutionary process. By the further optimization of the BP, the number of training cycles achieved the original maximum setting of 20,000, and an accuracy of 10^−3^ but not the target of 10^−4^ was reached.

### Model validation results

The changes of fitness in the cross-validation test are shown in Fig. 4. The RMSECV was 0.1398±0.0488 (n=6). The R of cross-validation between the true and predicted values was 0.9959±0.0027 (n=6). The comparison of true and predicted values of I_0_ is shown in Fig. 5. All the values of R are >0.99 and the prediction of the bitterness intensity is comparatively accurate.

### Final model

Regarding all data as a training set for modeling, the determination coefficient (R^2^) was 0.99965±0.00004 (n=4). A comparison of the results between the true and predicted values in the model and the standardized residuals is shown in Fig. 6. The results show that the model accurately predicted the bitterness intensity of unknown samples.

### MLR

The RMSECV was 0.7440. The R of cross-validation between the true and predicted values was 0.8957. Regarding all data as a training set for modeling, the constant term and the coefficients of ZZ, JE, BB, CA, GA, DA and AB in regression equation were 15.5297, −0.0009, 0.0055, 0.0000, −0.0235, −0.0029, 0.0047 and 0.0050, respectively. The R^2^ was 0.9896. The fitting charts are shown in Fig. 7A and B.

### PLS regression

The results showed that the modeling effect was the most accurate when the number of latent variables equaled five. The optimal RMSECV was 0.5273. The R of cross-validation between the true and predicted values was 0.9521. Regarding all data as a training set for modeling, the R^2^ was 0.9915. The fitting charts are shown in Fig. 7C–F.

### Artificial neural networks

In six parallel cross-validation tests, the RMSECV was 0.7253±0.1656. The R of cross-validation between the true and predicted values was 0.9011±0.0589. One of the comparisons is shown in Fig. 7 (R=0.9212). Regarding all data as a training set for modeling, the R^2^ was 0.9991±0.0002 (n=4) following four parallel trials. The fitting charts are shown in Fig. 7G and H.

### Comparison of several methods

The R values for the cross-validation between the true and predicted values for the four methods are compared in Fig. 8.

## Discussion

The present study established a BPM of berberine hydrochloride by combing a GA and a BPNN. Using the global optimization ability of the GA the parameters of the BPNN, such as initial weight, were optimized. The BPNN training function further optimized the parameters so that they were able to play to their advantages. The fitting degree of the model of the training set in this study was high (R^2^=0.99965), the RMSEVC in the cross-validation was 0.1398 and the R between the true and predicted values was 0.9959, suggesting that the modeling method is reliable and the model has satisfactory predictive ability. MLR and PLS regression have less accuracy than GA-BP as they are linear methods. BPNNs are non-linear, but easily fall into the local extreme point and are not superior to the GA-BP method.

Due to the correlation between the bitterness and concentration of drugs, it is possible to use the method used in this study to predict the concentration of drugs with the same system. The rational Weibull-logarithmic model has been established and reported in a previous study (20). This model is in line with the Weber-Fechner law (21), which is a law explaining the logarithmic association between taste intensity and taste stimulus in moderate stimulus conditions of the following formula: S = KlgR (22), where S is sensory intensity, R is stimulus intensity and K is the constant. The model is as follows: *I*_0_ = 1.5994 × log_10_ (c), where the unit of c (concentration) is μM (μmol/l) (R^2^ = 0.9665). A more accurately fitting model was used in the present study, which is a Weibull model (R^2^=0.9973, which is higher than that of the logarithmic model).

In conclusion, the BPM created in the present study, which is based on the e-tongue and GA-BP, may be used as a BPM for berberine hydrochloride of different concentrations. It also provides a reference for the generation of BPMs for other drugs. Additionally, the algorithm used in this study provides a rapid and accurate quantitative method for analyzing e-tongue data.

## Figures and Tables

**Figure 1:** Flow chart of the GA-BP. GA-BP, genetic algorithm-back-propagation neural network.

**Figure 2:** Concentration and corresponding rank bitterness intensity of the nine samples (S1–S9).

**Figure 3:** (A) Fitness curve of the GA and (B) training curve of the GA-BP. GA-BP, genetic algorithm-back-propagation neural network.

**Figure 4:** Fitness curve of the GA (cross-validation). GA, genetic algorithm.

**Figure 5:** Prediction values vs. the *I_0_* of the GA-BP (cross-validation). *I_0_*, rank bitterness intensity; GA-BP, genetic algorithm-back-propagation neural network.

**Figure 6:** (A) Prediction values of *I_0_* vs. the *I_0_* of the GA-BP and (B) standardized residuals of the GA-BP model. *I_0_*, rank bitterness intensity; GA-BP, genetic algorithm-back-propagation neural network.

**Figure 7:** Prediction values of *I_0_* vs. the *I_0_* of MLR, PLS regression and BPNN models and optimization of the number of latent variables in the PLS regression model. Prediction values for (A and B) MLR and (C and D) PLS regression. (E and F) Optimization of the number of latent variables in PLS regression. (G and H) Preduction values for the BPNN. *I_0_*, rank bitterness intensity; MLR, multiple linear regression; PLS, partial least squares; BPNN, back-propagation neural network; R, correlation coefficient; R^2^, determination coefficient; RMSECV, root mean square error of cross-validation.

**Figure 8:** R values (cross-validation) of the four methods. R, correlation coefficient; MLR, multiple linear regression; PLSR, partial least squares regression; BPNN, back propagation neural network; GA-BP, genetic algorithm-back-propagation neural network.

**Table I:** Bitterness rank and the concentration of the corresponding reference samples.

No.	Description of intensity of bitterness	Rank assigned	Scale	Concentration of reference samples mg/ml (mM)
1	Imperceptible	I	(0.5, 1.5)	0 (0)
2	Slight	II	(1.5, 2.5)	0.01 (0.027)
3	Moderate	III	(2.5, 3.5)	0.05 (0.134)
4	Great (but acceptable)	IV	(3.5, 4.5)	0.1 (0.269)
5	Extreme (almost unacceptable)	V	(4.5, 5.5)	0.5 (1.344)
